The article "Clinical Significance of Peripheral Blood Th1 and Th17 Cell Content and Serum IL-35 and IL-17 Expression in Patients with Ankylosing Spondylitis" was retracted in 2023. Reasons: unreliable results or conclusions; concerns about the data; concerns about the peer review; concerns about the citations.

# Clinical Significance of Peripheral Blood Th1 and Th17 Cell Content and Serum IL-35 and IL-17 Expression in Patients with Ankylosing Spondylitis

**DOI:** 10.1155/2022/6540557

**Published:** 2022-05-18

**Authors:** Haitao Tan, Shan Huang, Tingrui Wang

**Affiliations:** ^1^Department of Spinal Surgery, Hainan Province Clinical Medical Center, The First Affiliated Hospital of Hainan Medical University, Haikou, Hainan 570102, China; ^2^Department of Cardiology, The First Affiliated Hospital of Hainan Medical University, Haikou 570102, China

## Abstract

**Objective:**

To evaluate the clinical significance of peripheral blood T helper cell 1 (Th1) and T helper cell 17 (Th17) cell content and serum (interleukin) IL-35 and IL-17 expression in patients with ankylosing spondylitis (AS).

**Methods:**

In this retrospective study, we included and assigned 60 cases of AS patients enrolled in our hospital from January 2019 to January 2020 to an active group (ankylosing spondylitis disease activity score (ASDAS) ≥2.1, *n* = 28) and a static group (ASDAS<2.1, *n* = 32) according to the degree of disease activity. The logistic propensity score matching method was used to include 60 healthy individuals after a physical examination during the same period in the control group. The peripheral blood Th1 and Th17 cell content and the levels of serum IL-35 and IL-17 were determined and analyzed.

**Results:**

Statistically significant differences were found in the Th1 cell ratio and Th17 cell ratio between the control group and the other two groups (*P* < 0.05), and the static group yielded a higher Th1 cell ratio and a lower Th17 cell ratio than the active group (*P* < 0.05). Statistically significant differences were also observed in the serum IL-35 and IL-17 levels between the control group and the other two groups (*P* < 0.05), and the static group had a higher IL-35 level and a lower IL-17 level than the active group (*P* < 0.05).

**Conclusion:**

The imbalance of Th17/Th1 cell content of AS patients is characterized by high expression of IL-17 and low expression of IL-35. The increased activity of AS was associated with a dominant state of Th17 cells and a significant increase in IL-17 expression, indicating that Treg/Th17 imbalance is closely related to the development of AS, which may provide new ideas for the prevention and treatment of AS.

## 1. Introduction

Ankylosing spondylitis (AS) is an autoimmune disease with complex pathogenesis and insidious early symptoms. Approximately, 88% of patients first manifest as sacroiliac arthritis which may develop to the cervical spine lesion, and the rest 12% were primarily diagnosed with the cervical spine or the entire spine lesion [1–3], in which the axial bone joints and bone attachment points are severely damaged, resulting in severe inflammatory pain and even spinal flexion [4]. Recent reports have pointed out a close relation of the cause of AS to abnormal immune function. The study by Hoyt et al. confirmed an important correlation between CD4^+^T in T lymphocyte subsets and patient prognosis [5]. Specifically, the imbalance of T helper cell 1 (Th1), Treg, and T helper cell 17 (Th17), which exist in CD4^+^T, is the main contributory factor to the occurrence and development of AS. Moreover, there are also a series of related cytokines in Th1, Treg, and Th17, such as (interleukin) IL-17 and related inflammatory cytokines secreted by Th17 to exacerbate the autoimmune diseases [6–8]. The cytokine IL-35, secreted by Treg, can control the proliferation and differentiation of Treg and Th17 and regulate the expression level of IL-17 by influencing Th17, which is involved in immune-mediated diseases [9–11].

Inflammation is the key factor causing bone destruction and pathological ossification in AS patients. Repeated inflammation is associated with bone erosion and heterotopic ossification, leading to fusion and stiffness of the bone and joint, which restricts the patient's movement and seriously compromises daily life. Therefore, inflammation management is the key to deferring the course of AS and preventing disability. Th17 is a major effector cell in AS inflammation development and mediates AS inflammation through the characteristic secretion of cytokine IL-17, which induces proinflammatory mediators and chemokines. Therefore, inhibition of Th17 differentiation and reduction of IL-17 secretion are important targets for AS inflammation control. Transcription factors initiate Th17 cells to differentiate specific transcription factor retinoid-acid receptor-related orphan receptor yt (RORyt). There are many methylations of histone H3 at lysine27 (H3K27me3) markers in the promoter region of the upstream signaling molecule STAT3 and the gene encoding the downstream effector IL-17, and H3K27me3 plays an important regulatory role in the differentiation bias of Th17.

The exploration of the function of the cells and the expression of related cytokines may reap huge fruits in the monitoring of the changes in the patient's condition and the adjustment of the clinical treatment schemes. However, current research focuses more on the balance of Th1/Treg, yet few scholars have been able to draw on any systematic research into the clinical significance of the combination of Th17 with IL-17 and IL-35 in AS. Accordingly, this study is to evaluate the clinical significance of peripheral blood Th1 and Th17 cell content and serum IL-35 and IL-17 expression in patients with AS. The report is as follows.

## 2. Materials and Methods

### 2.1. General Information

In this retrospective study, we included and assigned 60 cases of AS patients enrolled in our hospital from January 2019 to January 2020 to an active group (ankylosing spondylitis disease activity score (ASDAS) ≥2.1, *n* = 28) and a static group (ASDAS<2.1, *n* = 32) according to the degree of disease activity. The logistic propensity score matching method was used to include another 60 healthy individuals after a physical examination during the same period in the control group. This study was approved by the Ethics Committee of the First Affiliated Hospital of Hainan Medical College, and the ethics approval number is 2018-11-12.

### 2.2. Diagnostic Criteria

(1) Duration of lower back pain lasts for at least 3 months, and the pain is relieved with activity but not by rest; (2) limited movement of the lumbar spine in anterior-posterior and lateral flexion directions; (3) thoracic gallery extension is smaller than normal for the same age and sex; (4) with bilateral sacroiliac arthritis grade II-IV, or unilateral sacroiliac arthritis grade III-IV. The diagnosis of AS is confirmed if the patient meets (4) and any of (1)–(3).

### 2.3. Inclusion Criteria

(1) The patients or their family members signed the informed consent form after being fully informed of the purpose and process of the study; (2) the patient was diagnosed with AS after examination, in line with the New York AS classification standard; human leukocyte antigen B27 was positive, and the course of the disease was more than 3 months [12, 13]; (3) the patient had no recent use of glucocorticoids or anti-rheumatic drugs [14, 15]; (4) aged over 18 years old; (5) the control group had no rheumatic diseases or other autoimmune diseases, with normal liver, kidney, and heart functions; (6) X-ray sacroiliac joint grading: grade 0: normal; grade I: suspicious changes; grade II: mild abnormalities, limited erosion and sclerosis, but no change in the joint space; grade III: obvious abnormalities, moderate or progressive skeletal iliac arthritis, with one or more of the following changes (erosion, sclerosis, widening or narrowing of the joint space, or partial ankylosis); grade IV: severe abnormalities, i.e., complete joint ankylosis.

### 2.4. Exclusion Criteria

(1) With mental problems that prevented communication; (2) with other organic diseases, combined with abnormal blood system conditions; (3) during pregnancy or lactation; (4) with acute and chronic infections; (5) with joint pain not caused by AS; (6) with other seronegative spondyloarthropathies; (7) with advanced spinal ankylosis and severe joint deformities; (8) with acute ophthalmia that requires hormone therapy; (9) with severe primary diseases such as cardiovascular, hematopoietic, and other systems.

### 2.5. Methods

The cell content of Th1 and Th17 in the peripheral blood and the levels of IL-35 and IL-17 in the serum of the research subjects were determined. The specific steps were as follows: (1) Th1 and Th17: (1) 5 ml of morning fasting venous blood from the patients was collected, placed in a heparin sodium anticoagulation tube, diluted with an equal volume of phosphate buffer solution, and then centrifuged with human lymphocyte separator to obtain mononuclear cells. The cell concentration was then adjusted to 2 × 106/ml and inoculated in a six-well culture plate, with phorbol ethyl ester, ionomycin, and monensin added to the wells, and the plate was placed in a 37°C, 5% carbon dioxide cell incubator for 5 hours. (2) A measuring tube and an isotype control tube were set according to the cell count, and then phycoerythrin-labeled mouse anti-human CD8 monoclonal antibody and phycoerythrin-cyanine dye-labeled mouse anti-human CD3 monoclonal antibody were added and incubated at 5°C for 0.5 h. (3) At room temperature, the fixation buffer was added and rested for 10 minutes without light followed by centrifugation. After the removal of the supernatant, the plate was rinsed with phosphate buffer solution, prior to the use of permeabilization wash buffer for the staining of the intracellular cytokines. (4) IL-17A-FITC and IFN-*γ*-FITC were added to the assay tube for staining, with the control tube for isotype control, incubated at 5°C for 0.5 h, and rinsed with phosphate buffer solution, to suspend the cells in phosphate buffer solution. (5) Th1 and Th17 were detected by flow cytometry (Aisen Bio-Hangzhou Co., Ltd., Zhejiang Food and Drug Administration Zhunzi 2014 no. 2400581). The above kits were purchased from Shanghai Ruibosai Biotechnology Co., Ltd. (2) IL-35 and IL-17: 5 ml of morning fasting venous blood was collected from the patients and placed in a vacuum blood collection tube, followed by the centrifugation at 4000 r/min for 15 minutes to separate the serum. The levels of IL-35 and IL-17 were determined by the enzyme-linked immunosorbent assay (Beijing Kewei Clinical Diagnostic Reagent Co., Ltd., S20060028), and the operation steps complied strictly with the kit instructions.

### 2.6. Observational Indexes

The ratio of Th1 and Th17 cells in the peripheral blood and the level of serum IL-35 and IL-17 were compared.

### 2.7. Statistical Processing

In this research, the data were processed by SPSS20.0, and GraphPad Prism 7 (GraphPad Software, San Diego, USA) was used to plot the graphics. The K-S test was used to examine the normality of the data. The research included the count data and measurement data. A *t*-test was adopted for the analysis of the measurement data which were represented by ($\bar{x}$ ± *s*), and an *X*^2^ test was used for analyzing the count data which were expressed as (n (%)). *P* < 0.05 indicated that the difference was statistically significant.

## 3. Results

### 3.1. Comparison of Baseline Data

There were statistical differences in the ASDAS, erythrocyte sedimentation rate, and C-reactive protein levels of the research subjects (*P* < 0.05), and no statistical differences in other general data (*P* > 0.05) (see Table 1).

### 3.2. Comparison of Th1 and Th17 Cell Ratios in Peripheral Blood

Statistically significant differences were found in the Th1 cell ratio and Th17 cell ratio between the control group and the other two groups (*P* < 0.05), and the static group yielded a higher Th1 cell ratio and a lower Th17 cell ratio than the active group (*P* < 0.05) (see Table 2, Figure 1, and Figure 2).

### 3.3. Comparison of Serum IL-35 and IL-17 Levels

Statistically significant differences were detected in the serum IL-35 level and serum IL-17 level between the control group and the other two groups (*P* < 0.05), and the static group was observed a higher IL-35 level and a lower IL-17 than the active group (*P* < 0.05) (see Table 3, Figure 3, Figure 4).

## 4. Discussion

AS is an autoimmune disease that mainly affects the sacroiliac joints and axial bone joints of the patient with elusive pathogenesis. It was believed that the main cause of AS is heredity, in which infection and immunity are considered the main contributory factors [16]. Recent studies have confirmed that abnormal immune response triggered by abnormal differentiation of T lymphocyte subsets is the major cause of AS [17]. Specifically, CD4^+^T, containing Th1, Treg, Th17, and other related cells, is the main lymphocyte in the T lymphocyte subset that affects the development of autoimmune diseases. Th1, secreting IL-2, TNF-*β*, and other cytokines can induce cellular immune responses such as AS, which is secondary to the body's abnormal regulatory effect after an inflammatory response [18]. The report of Monasterio et al. pointed out a decreasing trend of Th1 in patients with static rheumatoid arthritis, with a lower Th1 cell content than that of patients in an active phase [19]. The present study revealed a higher Th1 cell content in the static group than that in the active group, which may be attributed to the migration of Th1 cells in large numbers after the suppression of the immune effect mediated by Th1 during the active phase. The increase in the Th1 ratio indicates that the Th1 content commences to levels off within a normal range along with the improvement of the patient's condition.

The balance between Treg, Th17, and Th1 in peripheral blood of AS patients and their association with disease activity have been investigated at the cellular and genetic levels to provide new ideas for the prevention and treatment of AS. The aberrant differentiation of Th17 cells mediates AS inflammation and is the central effector cell triggering AS inflammation [15]. IL-17 is highly expressed in the serum and tissues of patients with various autoimmune diseases, such as rheumatoid arthritis, systemic lupus erythematosus, multiple sclerosis, and ankylosing spondylitis [19–23], and is closely related to the pathogenesis of autoimmune and inflammatory diseases. The significantly decreased level of H3K27 trimethylation in peripheral blood mononuclear cells (PBMC) of AS patients compared with normal individuals may be one of the important mechanisms that activate the characteristic Th17 transcription factor RORc and the upstream JAK/STAT signaling pathway, mediating the inflammation of AS.

The changes of Th1 result in the imbalance of Th1/Th17, prior to the occurrence or intensification of AS. Th17, a key factor affecting autoimmune diseases, can promote the secretion of IL-17 which is a proinflammatory cytokine that mediates the inflammatory response. Studies have stated a high expression of IL-17 in lupus erythematosus, rheumatoid arthritis, and other relevant diseases and a positive correlation between IL-17 and the severity of the diseases, which demonstrate a close relationship between the above-mentioned autoimmune diseases and IL-17 [21, 22]. In the present study, the Th17 level of the active group was higher than that of the static group and the control group, with a drastically increased IL-17 level in the active group, indicating a synergistic effect of Th17 and IL-17 in terms of the pathogenesis of AS. Therefore, the monitoring of Th17 and IL-17 levels in clinical practice and the targeted Th17 differentiation to control the secretion of IL-17 predominantly contribute to the prevention of AS from further aggravation.

According to the latest research, IL-35, as an important indicator in regulating Th17 differentiation, can reverse the imbalance of Th1/Th17 and regulate the secretion of IL-17 [23]. The research of Lee and Song. pointed out that the transfer of IL-35 in the collagen-induced mouse joint model can enhance the stability of CD4^+^T and inhibit the abnormal proliferation of CD4^+^ cells, thereby mitigating the inflammatory response and alleviating the symptoms of arthritis in mice [24]. In the present study, statistically significant differences were detected in the serum IL-35 level and serum IL-17 level between the control group and the other two groups (*P* < 0.05), and the static group showed a higher IL-35 level than the active group (*P* < 0.05). The research of scholar Maksymowych et al. further proved a negative correlation of IL-35 with erythrocyte sedimentation rate and C-reactive protein level [25], indicating the impact of the high expression of IL-35 on the inflammatory response in patients. Accordingly, in addition to the inhibitory effect of IL-35 on the inflammatory level of AS patients, IL-35 can also regulate Th17, IL-17, and other related indicators, to achieve a promising clinical treatment effect. Nonetheless, It is worth noting that the exact regulatory mechanism of IL-35 on AS is still unclear, which requires further research for clarification.

The innovation of this study is that the presence of dysregulated Th17/Th1 cell balance and reduced expression of IL-17 and IL-35 in AS patients are closely related to AS disease activity, which may provide new ideas for the prevention and treatment of AS. Immediate intervention or treatment should be given at the early stage of multi-indicator alterations to avoid persistent deterioration of AS. The limitation of this study is the absence of joint testing of the diagnostic efficacy of multiple indicators, which will be further investigated in future studies.

In conclusion, the imbalance of Th17/Th1 cell content of AS patients is characterized by high expression of IL-17 and low expression of IL-35, which are significantly correlated with the activity of AS, showing great potential in monitoring the development of AS.

The horizontal axis of Figure 1 from left to right is the control group, the active group, and the static group, and the vertical axis is the ratio of CD4^+^IFN-*γ* + Th1 cells (%). The Th1 cell ratio of the control group was significantly higher than that of the active group (8.10 ± 1.21 vs 4.21 ± 1.10, *P* < 0.05) and the static group (8.10 ± 1.21 vs 7.21 ± 1.26, *P* < 0.05). The Th1 cell ratio of the static group was significantly higher than that of the active group (7.21 ± 1.26 vs 4.21 ± 1.10, *P* < 0.05).

The horizontal axis in Figure 2 from left to right is the control group, the active group, and the static group, and the vertical axis is the ratio of CD4 + IL-17 Th17 cells (%). The Th17 cell ratio of the control group was significantly lower than that of the active group (0.39 ± 0.09 vs 1.68 ± 0.19, *P* < 0.05) and the static group (0.39 ± 0.09 vs 0.62 ± 0.10, *P* < 0.05). The Th17 cell ratio of the static group was significantly lower than that of the active group (0.62 ± 0.10 vs 1.68 ± 0.19, *P* < 0.05).

The dotted line in Figure 3 is the control group, the square line is the active group, the triangle line is the static group, and the vertical axis is the serum IL-35 level (pg/ml). The serum IL-35 level of the control group was significantly higher than that of the active group (45.26 ± 15.64 vs 15.98 ± 3.68, *P* < 0.05) and the static group (45.26 ± 15.64 vs 30.21 ± 6.98, *P* < 0.05). The level of serum IL-35 in the static group was significantly higher than that in the active group (30.21 ± 6.98 vs 15.98 ± 3.68, *P* < 0.05).

The dotted line in Figure 4 is the control group, the square line is the active group, the triangle line is the static group, and the vertical axis is the serum IL-17 level (pg/ml). The serum IL-17 level of the control group was significantly lower than that of the active group (7.98 ± 1.11 vs 40.26 ± 4.22, *P* < 0.05) and the static group (7.98 ± 1.11 vs 13.98 ± 1.59, *P* < 0.05). The serum IL-17 level of the static group was significantly lower than that of the active group (13.98 ± 1.59 vs 40.26 ± 4.22, *P* < 0.05).

## Figures and Tables

**Figure 1:** Comparison of the ratio of CD4^+^IFN-*γ*+Th1 cells (*x* ± *s*,%).

**Figure 2:** Comparison of the ratio of CD4^+^IL-17 Th17 cells (*x* ± *s*, %).

**Figure 3:** Comparison of serum IL-35 levels (*x* ± *s*, pg/ml).

**Figure 4:** Comparison of serum IL-17 levels (*x* ± *s*, pg/ml).

**Table 1:** Comparison of general information of research objects.

Groups	Active group (n = 28)	Static group (n = 32)	Control group (n = 60)	*P* value
Gender				>0.05
Male	25	28	54	
Female	3	4	6	
Age (year)				
Age range	21−46	22−47	22−46	
Mean age	30.22 ± 5.24	30.29 ± 5.23	30.26 ± 5.14	>0.05
Course of disease (year)	2.75 ± 1.21	2.72 ± 1.02	—	>0.05
ASDAS (points)	4.10 ± 1.22	1.68 ± 0.31	—	<0.05
Erythrocyte sedimentation rate (mm/h)	45.98 ± 15.32	11.26 ± 1.10	18.21 ± 2.20	<0.05
C-reactive protein (mg/L)	22.68 ± 15.11	5.98 ± 2.68	2.12 ± 0.54	<0.05
Living habits				>0.05
Smoking	24	27	50	
Drinking	25	28	52	
Underlying disease				>0.05
Hypertension	15	23	—	—
Diabetes	12	20	—	—
Education level	—	—	—	>0.05
Middle school and below	8	10	20	—
High school	15	17	30	—
Junior college and above	5	5	10	—
Monthly income (yuan)				>0.05
≥3000	18	22	42	
＜3000	10	10	18	

**Table 2:** Comparison of Th1 and Th17 cell ratios in peripheral blood.

Groups	n	Th1 (%)		Th17 (%)	
		Mean value	Sd	Mean value	Sd
Control group	60	8.10	1.21	0.39	0.09
Active group	28	4.21	1.10	1.68	0.19
Static group	32	7.21	1.26	0.62	0.10

**Table 3:** Comparison of serum IL-35 and IL-17 levels.

Groups	n	IL-35 (pg/ml)		IL-17 (pg/ml)	
		Mean value	Sd	Mean value	Sd
Control group	60	45.26	15.64	7.98	1.11
Active group	28	15.98	3.68	40.26	4.22
Static group	32	30.21	6.98	13.98	1.59

## Data Availability

The data are available upon request from the corresponding author.
